RETRACTED

# Liver Protection Mechanism and Absorption Promotion Technology of Silybin Based on Intelligent Medical Analysis

**DOI:** 10.1155/2021/9968016

**Published:** 2021-07-03

**Authors:** Bingbing Yan, Chuanying Zhang

**Affiliations:** ^1^Pharmacy, Guangrao People's Hospital, Dongying 257300, Shandong, China; ^2^Zhucheng People's Hospital, Zhucheng 262200, Shandong, China

## Abstract

With the continuous popularization of smart medicine, the protective effect of silibinin in the liver has attracted much attention. This study mainly explores the liver protection mechanism and absorption promotion technology of silybin based on intelligent medical analysis. Refining of silibinin: accurately weigh 1.0 g of silibinin in a three-necked flask; gradually add 50 mL of anhydrous methanol, reflux and filter the precipitated solid; and weigh it after drying. ICR male mice were taken as experimental subjects and randomly divided into groups of 10 each. The mice in the normal group and the model group were given intragastrically with 0.5% CMC-Na solution; the mice in the silibinin group were given intragastrically with SB/CMC-Na suspension; the mice in the remaining groups were given low, medium, and high-dose suspensions to their stomachs, and silibinin 23 acylate/CMC-Na suspension was administered at a dose of 10 mL/kg for 7 consecutive days. After that, the mice were fasted for 12 hours. After 6 hours of fasting (18 hours after modeling), the blood cells from their orbits were taken, placed in a 37°C water bath for 30 minutes, and centrifuged at 4000 rpm for 10 minutes, and then the serum was taken; the activity equivalent of AST and ALT in serum was measured; serum determination Medium AST and ALT vitality. The mice were killed by decapitation, fresh liver tissue was immediately collected, and part of it was frozen in liquid nitrogen for the RT-PCR test. The hepatocyte expansion and death were observed using a transmission electron microscope, and the oncosis index (OI) was calculated. Another part of the liver tissue was fixed in 4% paraformaldehyde solution, embedded in paraffin, dehydrated, and sliced at 4 *μ*m. Some sections were stained with conventional HE, and the pathological changes of liver cells were observed under light microscope; some sections were subjected to immunohistochemistry. Only one mouse died when 240 mg/kg of silibinin was given 10 minutes after the model was modeled. However, when 240 mg/kg silibinin was given to the mice 20 minutes after modeling, the mortality rate of the mice rose to 50%, and the therapeutic effect was significantly weakened. This research is helpful to advance the research of silybin in liver protection.

## 1. Introduction

Fast-paced life and increasingly serious environmental pollution have caused various diseases, and human health is seriously threatened. Timely and accurate disease diagnosis and treatment are very important. However, due to the limitation of regional economic development, the distribution of medical resources in various regions is extremely uneven. Missing the best time for treatment and misdiagnosis of the disease may cause the patient to suffer unbearable consequences. In order to improve the accuracy of diagnosis, more and more advanced medical equipment inspections are used in hospitals. Doctors can diagnose diseases more accurately through clear and objective data in the inspection results.

RETRACTED

Some swelling-like cell deaths often occur during acute liver cell injury. Due to differences and deficiencies in understanding, this type of cell death has been simply described as turbidity and swelling in the past. Patients with functional gastrointestinal diseases often have physical symptoms, which affect their quality of life to a certain extent, and cause a great burden on their economic and social life.

Although a large number of experiments have been conducted on allergic hepatitis using animal models, it is still difficult to draw pictures of chronic hepatitis. Ali et al. conducted this research to introduce an animal model that approximates the chronic mechanism of human hepatitis. The study also aims to examine the hepatoprotective effects of curcumin, silybin phytosome®, and *α*-R-lipoic acid on thioacetamide (TAA)-induced hepatitis in mice. TAA was administered intraperitoneally at a dose of 200 mg/kg 3 times a week for 4 weeks. At the end of this period, a group of mice was killed to assess the occurrence of chronic hepatitis compared with the corresponding control group. TAA administration was then discontinued, and the remaining animals were divided into four groups. Group 1 was untreated, while groups 2–4 received oral curcumin every day. Their research only grouped the animals and did not further discuss the results of the research [1]. Tereshchenko et al. believe that silybin (Slb) and ursodeoxycholic acid (UDCA) are hepatoprotective agents used in the treatment of liver and biliary pathology. However, the low bioavailability of these drugs limits their applications. To solve this problem, they incorporated Slb and UDCA into a polymer carrier based on polylactic acid and poly (lactic acid-co-glycolic acid) through nanoprecipitation. The polymer form they obtained according to the method developed and optimized is nanoparticles with a size of 100 to 200 *μ*m. Although their research in vitro shows that the hepatoprotective activity of polymer nanoparticles containing Slb and UDCA is 1.5–2 times higher than that of free substances, the research lacks contrast [2]. Federico et al. compare silibinin with phosphatidylcholine (Realsil) (*R*) or placebo (*P*) combined with silibinin in the serum of nonalcoholic steatohepatitis (NASH) patients treated for 12 months (T 12). According to the oxidative stress index level, the expression effect of oxidative stress in human endothelial cells after the adjustment of the patient's serum is studied. They recruited 27 histological NASH patients. They also measured human endothelial cells in the serum of patients exposed or not exposed to H2O2. At *T* 12, alanine aminotransferase (*p*=0.038), transforming growth factor-*β* (*p*=0.009), and procollagen I (*p*=0.001) decreased. By dividing patients into two groups, compared with *T* 0, (PI/RI) increase (TB/RS) (P-II/R-II) at *T* 12 decreases. Although their research can confirm that the CAT activity of conditional endothelial cells increases at T12 in the two groups (*p* 0.05 and *p*=0.001, respectively), the accuracy of the research is not high [3]. Belli et al. believe that the oral multi-kinase inhibitor Regorafenib has shown a survival benefit in patients with metastatic colorectal cancer (mCRC) who have progressed after all standard therapies. However, new strategies to improve tolerance and enhance anti-cancer efficacy are needed. They have evaluated the effects of regorafenib in combination with silybin (a biologically active ingredient extracted from the seeds of milk thistle) in a group of human colon cancer cells in vitro. In addition, they prospectively treated 22 patients with refractory mCRC with regofinil plus silibinin. Although regorafenib treatment in their study determined a dose-dependent growth inhibitory effect, and silibinin treatment had no antiproliferative effect in all cancer cells tested, the level of intracellular reactive oxygen species was not studied [4].

RETRACTED

As the digestive gland outside the human gastrointestinal tract, the liver is closely related to the digestion and absorption function of the gastrointestinal tract. The gastrointestinal tract is the earliest and most severe extrahepatic organ affected by liver disease; gastrointestinal dysfunction can also affect the repair of liver injury, and even aggravate the damage process. Refining of silibinin: accurately weigh 1.0 g of silibinin in a three-necked flask, gradually add 50 mL of anhydrous methanol, reflux, filter the precipitated solid, and weigh it after drying. ICR male mice were taken as experimental subjects and randomly divided into groups of 10 each. The mice in the normal group and the model group were given intragastrically 0.5% CMC-Na solution; the mice in the silibinin group were given intragastrically SB/CMC-Na suspension; the remaining groups of mice were given intragastrically low, medium, and high doses, and silibinin 23 acylate/CMC-Na suspension was administered at a dose of 10 mL/kg for 7 consecutive days. After that, the mice were fasted for 12 hours without water; 6 hours later (18 hours after modeling), blood was taken from the orbit and placed in a 37°C water bath for 30 minutes, centrifuged at 4000 rpm for 10 minutes, and then the serum was taken; serum determination Medium AST and ALT vitality. The mice were killed by decapitation, fresh liver tissue was immediately collected, and part of it was frozen in liquid nitrogen for the RT-PCR test. The hepatocyte expansion and death were observed by transmission electron microscope, and the oncosis index (OI) was calculated. Another part of the liver tissue was fixed in 4% paraformaldehyde solution, embedded in paraffin, dehydrated, and sliced at 4 *μ*m. Some sections were stained with conventional HE, and the pathological changes of liver cells were observed under light microscope; some sections were subjected to immunohistochemistry. This research is helpful to advance the research of silybin in liver protection.

## 2. Liver Protection Mechanism of Silybin

### 2.1. Silybin

Silymarin has been used to treat hepatitis and liver cirrhosis for more than two thousand years. Studies have shown that silymarin can prevent liver damage caused by CCl4, galactosamine, alcohols, and other liver toxins (such as Amanita phalleodes). Its mechanism of action is mainly concerned with the aspects of anti-liver fibrosis, protection of liver cells, promotion of repair and regeneration of liver cells, anti-lipid peroxidation, and immunomodulatory effects. In Wistar male mice, injection of CCl4 mineral oil solution leads to cirrhosis and diffuse necrosis. Silymarin has a significant inhibitory effect in the thinning of collagen bands and decreased liver collagen content, etc. It can also inhibit the increase in blood ALT, ALP, and total bilirubin caused by CCl4 [5, 6]. Silybin (Sb) is the main flavonoid in milk thistle extract. It is used to treat various acute and chronic liver toxicity, inflammation, fibrosis, and oxidative stress. Many studies have shown that Sb is also active against different cancers, and it has recently been suggested that it is beneficial to patients with type 2 diabetes. However, Sb is a compound with low water solubility and low permeability [7]. The molecular structure of silybin is shown in Figure 1.

The presence of flavonoid nucleus, benzodioxane structure, and polyhydroxyl groups in the silibinin molecule are all beneficial to the improvement of hepatoprotective activity. The 3-hydroxyl and 23-hydroxymethyl groups are necessary to maintain the activity. Assigned to a certain cluster center *Cj* (0 < *j* < *k*) [8].

(1) $$\begin{array}{c} \left\|x_{i}-C_{j}\right\|=\min\left\|x_{i}-C_{l}\right\|. \end{array}$$

Calculate the new vector value *C*_*j*_ of each cluster center.

(2) $$\begin{array}{c} C_{j}={\left[C_{j1},C_{j2},...,C_{jp}\right]}^{\text{T}}. \end{array}$$

In the formula, *p* is the number of data attributes [9].

(3) $$\begin{array}{c} C_{jp}=\frac{1}{Nj}\underset{x\in s_{j}}{\sum }x\left(j=1,2,...,k\right). \end{array}$$

Adjust the series by dividing the *k* column to ensure that the evaluation scores of all series are within the interval (0, 1) [10, 11]. Let |*T*| be the sample size of data set *T*:

(4) $$\begin{array}{c} M\left(T\right)=-\overset{k}{\underset{i=1}{\sum }}\left(\left(\frac{\text{freq}\left(C_{i},T\right)}{\left|T\right|}\right)*\;\log_{2}\left(\frac{\text{freq}\left(C_{i},T\right)}{\left|T\right|}\right)\right). \end{array}$$

The data set *T* is split according to the attribute *V*, and the expected information calculation formula is [12]:

(5) $$\begin{array}{c} f\left(X_{i}\left(k\right)\right)=\frac{X_{i}\left(k\right)}{A\left(k\right)},\\ X_{\text{i}}=\left(X_{1i},X_{2i},\cdots ,X_{ji}\right),\\ i=1,2,\ldots ,n. \end{array}$$

According to the results of the evaluation, a judgment matrix of *n* evaluation indexes can be obtained, among which *C*1, *C*2, *C*3 … *Cn* is the evaluation index of medical APP user experience [13, 14].

(6) $$\begin{array}{c} M={\left(A_{ij}\right)}_{m\times n}=\begin{array}{c} C1\\ C2\\ \vdots \\ Cn \end{array}\left[\begin{array}{cccc} A_{11} & A_{12} & \cdots & A_{1n}\\ A_{21} & A_{22} & \cdots & A_{2n}\\ \vdots & \vdots & \vdots & \vdots \\ A_{n1} & A_{n2} & \cdots & A_{nn} \end{array}\right]. \end{array}$$

RETRACTED

### 2.2. Liver Protection

The liver is the central organ that stores carbohydrates and has the function of maintaining a relatively stable and even distribution of blood sugar. At the same time, it is also the main place for triglycerides, phospholipids, cholesterol metabolism, protein synthesis, and the “inactivation” of many hormones. It is responsible for the detoxification of human body toxins, the storage of nutrients, and the metabolism of multiple vitamins. It is one of the main organs of the human body. However, the effect of SIL on hepatocyte swelling and death is currently seldom studied, and its exact mechanism is still unclear. Drug-induced liver injury is an important part of toxicology research. Traditional in vivo tests have some shortcomings in the study of drug-induced liver damage. For example, it is difficult to distinguish between primary liver damage and secondary liver damage. Animal tests have disadvantages such as being time-consuming, large number of animals, and high cost. Compared with in vivo tests, in vitro tests can not only control environmental factors but also exclude the influence of interacting systems such as immune and neuroendocrine systems. It is faster and more economical, and has fewer errors between tests. In the current research of Silybum marianum against liver damage, the experimental drugs mostly use silybin as a single component, ignoring the other two main components in silymarin. The liver is the main site for drug metabolism. The liver parenchymal cells have a complete drug metabolism enzyme system and are the main site for drug biotransformation. Therefore, in vitro culture of hepatocytes plays an increasingly important role in liver disease research. Primary hepatocytes are often used in the study of drug metabolism in vitro. Primary hepatocytes cultured in vitro have many unique advantages: a large number of samples with relatively uniform characteristics can be obtained at the same time; the culture system contains only parenchymal cells, which is convenient for artificial control of culture conditions and eliminates the interference of many complicated factors; basically retains the liver. Some metabolic functions and cell differentiation states have a long survival time; the new method allows the measurement of drug concentration in cells and even organelles [15].

Inflammatory cytokines play an important role in the process of carbon tetrachloride liver injury. TNF-*α* and IL-1a show an increasing trend during the injury process, and immune neutralization can reduce the injury within a period of time. Others have also confirmed that TNF-*α* is very important in the process of liver injury, but the function of regulating the toxicity of acetaminophen is still controversial. Mice knocking out TNF-*α* are not immune to acetaminophen liver damage. IL-10 is another important cytokine, which can protect the liver by controlling the formation of NO and iNOS. Migration inhibitory factor (MIF) is a protein with the characteristics of cytokines, hormones, and enzymes. It promotes the production of other proinflammatory factors and adhesion molecules during the process of acetaminophen liver injury. MIF knockout mice are not sensitive to acetaminophen and can reduce IFN-Y and increase the expression of heat shock proteins. Heat shock proteins can combat many physiological and environmental stressors. Cyclooxygenase-2 can be used as a liver protective agent, which may be related to the enhanced expression of heat shock proteins. The importance of the project *C*_*i*_ relative to *C*_*j*_ can be expressed as [16, 17]:

(7) $$\begin{array}{c} a_{ij}=\frac{w_{i}}{w_{j}}. \end{array}$$

Its determinant can be expressed as

(8) $$\begin{array}{c} A=\left[\begin{array}{ccc} \frac{w_{1}}{w_{1}} & \cdots & \frac{w_{1}}{w_{n}}\\ \vdots & \vdots & \vdots \\ \frac{w_{n}}{w_{1}} & \cdots & \frac{w_{n}}{w_{n}} \end{array}\right],\\ W=\left[\begin{array}{c} w_{1}\\ \cdots \\ w_{n} \end{array}\right]. \end{array}$$

Therefore:

(9) $$\begin{array}{c} w_{i}=\frac{1}{n}\overset{n}{\underset{j=1}{\sum }}\frac{a_{ij}}{\sum_{i=1}^{n}a_{ij}},\;i,j=1,2,3\ldots n. \end{array}$$

RETRACTED

### 2.3. Smart Medical

Limited by the doctor's clinical experience and insufficient diagnosis and treatment skills, doctors find it difficult to identify cancer characteristics and make correct diagnoses at an early stage, and even produce serious consequences that delay the best treatment time. This situation is particularly obvious in primary medical institutions [18]. Therefore, how to improve the diagnosis, treatment level, and work efficiency of doctors for major diseases such as cancer and minimize the misdiagnosis and missed diagnosis of primary medical institutions has become a common goal globally [19]. In recent years, with the integration and penetration of new-generation information technologies such as big data and artificial intelligence with medical and health management, major developed countries have successively built a large number of intelligent medical detection systems in the fields of cancer diagnosis and treatment, serious cardiovascular and cerebrovascular disease risk warning, and chronic disease management. The medical auxiliary diagnosis system plays an important role in comprehensively improving the doctor's diagnosis and treatment capabilities. After years of construction and reform in China's medical and health industry, the level of medical services has been significantly improved, but the lack of high-quality medical resources has led to the inability to get a balanced distribution of resources, and a gap exists in the level of medical services between regions and between urban and rural areas. The emergence of intelligent medical auxiliary diagnosis system has brought new breakthroughs for improving the diagnosis and treatment capabilities of doctors at the grassroots level, narrowing the medical service gap between regions, and improving the overall medical service level of hospitals in China. However, in reality, the intelligent medical auxiliary diagnosis system has difficulties in deployment and insufficient popularization and application. How to make targeted improvements to the research and promotion of intelligent medical auxiliary diagnosis decision-making methods and systems has become a key issue in improving the level of medical services. *W* in the matrix is the eigenvector of *A*, then [20, 21]:

(10) $$\begin{array}{c} C\mathrm{.I}=\frac{\lambda_{\text{max}}-n}{n-1}. \end{array}$$

The smaller the *C.I* value, the higher the consistency. When the order is the same, the ratio of *C.I* to *C.R* is called the consistency ratio [22].

(11) $$\begin{array}{c} \text{C}.\text{R}=\frac{C\mathrm{.I}}{R\mathrm{.I}}. \end{array}$$

The uneven distribution of high-quality medical resources has led to a huge gap in medical services between urban and rural medical institutions, which is not conducive to the improvement of the overall medical level [23, 24]. At the same time, major diseases such as cancer have become a major obstacle to people's life extension in the new century, seriously threatening the lives and health of people globally [25]. People are eager to strengthen the diagnosis and treatment ability of doctors through technology and other means, especially the inexperienced doctors. The rapid development of artificial intelligence technologies such as deep learning has brought new hope and means for people to solve the above problems [26, 27]. The outstanding performance of these technologies in disease diagnosis and other aspects impressed people, and a large number of researchers have invested in the research, development, and application of intelligent medical auxiliary diagnostic systems to improve the diagnosis, treatment capabilities, and work efficiency of doctors, and narrow the gap in medical services between regions. All the weight results that pass the consistency test are clustered into groups, and the final weight coefficient *w*_*i*_^*G*^ of each indicator is obtained [28, 29]. The diagnosis process of a disease needs to consider a variety of complex factors. In order to dig out detailed disease diagnosis information, most intelligent medical systems start with a certain type of disease for targeted research, and collect multiple related factors of the disease to improve the accuracy of the final diagnosis. As in the past, each disease will have its own different system, which will lead to its poor applicability and inability to function. In the real diagnosis scenario, the patient himself or herself is often unable to determine which disease he or she is suffering from. The doctor first needs to ask various questions to determine the scope of the disease, supplemented by medical examination items, and finally diagnose the disease. Unlike most intelligent diagnosis systems that directly diagnose through existing information, the actual diagnosis process is often completed by continuously mining new information and gradually narrowing the scope of candidate diseases. It has good interpretability, and doctors also need to deal with encounters. For questions about patients, consult and search for the latest research progress or similar medical records. Therefore, how to apply artificial intelligence technology to realistic and complex diagnosis scenarios, assist doctors in disease diagnosis and at the same time help doctors accumulate medical experience and improve the level of medical treatment will have very important research significance.

(12) $$\begin{array}{c} w_{i}^{G}={\overset{K}{\underset{k=1}{\prod }}\left[w_{i}^{k}\right]}^{a_{k}},\;i=1,2,\ldots ,n. \end{array}$$

Due to the complex structure of the liver and the high noise of ultrasound images, it is not realistic to simply classify the data by the original gray value. So here, instead of using the commonly used piecewise function method to set the color value of the data, the value preprocessed with the original grayscale on each point is directly assigned to each point as its color value, so that the drawing can be made. The result is more detailed. Since the main target to be visualized is the part with higher gray, the original gray value is relatively low, and the opacity of the part as the background is set to its gray value and divided by *n*, and the gray value is higher. Set the partial opacity to 1.

(13) $$\begin{array}{c} X_{i}=\frac{\left(Hu_{\left(1,j,k\right)}-Hu_{\left(1,j,k\right)}\right)}{a}. \end{array}$$

Among them, *X*_*i*_ represents the degree of absorption of the small intestine under the influence of the liver.

RETRACTED

## 3. Liver Protection and Absorption Promotion Experiment

### 3.1. Experimental Animals

ICR mice (male), weighing 20 ± 2 g. The experimental animals were raised in a prescribed environment to ensure sufficient water source, 12/12 hour day/night, humidity 55 ± 5%, temperature 23°C, and fed with commercial feed.

### 3.2. Refining of Silybin

The purity of commercially available silybin is only 88%–89%, so it needs to be refined. Silybin has the highest solubility in methanol. Therefore, we refined it by recrystallization from anhydrous methanol, and measured its content by reversed-phase high-performance liquid method.

Operation method: precisely weigh 1.0 g of silibinin in a three-necked flask, gradually add 50 mL of anhydrous methanol, reflux for several hours, cool to room temperature with the oil temperature, and then stand in a refrigerator at 2°C. The precipitated solid was filtered and weighed 0.75 g after drying. The yield was 75%; its content was determined to be 98%.

### 3.3. Experimental Process

ICR male mice were used as experimental objects, and they were randomly divided into groups, 10 in each group: normal group, model group (CCl4 injury group), positive control group (a mixture injected with 200 mg/kg silibinin at a concentration of 20 mg/mL), silibinin 23 acylate low-dose group (100 mg/kg, concentration of 10 mg/mL suspension), silibinin 23 acylate middle-dose group (200 mg/kg, concentration 20 mg/mL suspension), silibinin 23 acylate high-dose group (300 mg/kg, 30 mg/mL suspension), and 300 mg/kg silibinin 23 acylate group (this group was only administered a suspension with a concentration of 30 mg/mL without modeling). The mice in the normal group and the model group were given intragastrically 0.5% CMC-Na solution; the mice in the silibinin group were given SB/CMC-Na suspension by intragastric administration; the mice in the other groups were given low, medium, and high doses. In the stomach, silibinin 23 acylate/CMC-Na suspension was administered at a dose of 10 mL/kg for 7 consecutive days. Two hours after gavage on the 7^th^ day, mice in the normal group and 300 mg/kg silibinin 23 acylation product group were injected intraperitoneally with soybean oil, and mice in the model group, positive control group, and low, medium, and high dose groups were injected intraperitoneally CCl4/soybean oil solution (CCI4 content is 0.25%), the dosage is 10 mL/kg. After that, the mice were fasted for 12 hours without water; 6 hours later (18 hours after modeling), blood was taken from the orbit and placed in a 37°C water bath for 30 minutes, centrifuged at 4000 rpm for 10 minutes, and then the serum was taken; serum determination Medium AST and ALT vitality.

### 3.4. Retention and Pathological Examination of Liver Tissue

The mice were killed by decapitation, fresh liver tissues were immediately collected, and part of it was frozen in liquid nitrogen for the RT-PCR test; some were cut into approximately 1 mm^3^ tissue pieces, quickly put into 2.5% glutaraldehyde fixative solution, and sent to the center of electron microscopy. Transmission electron microscope was used to observe the expansion and death of liver cells and calculate the oncosis index (OI). Another part of the liver tissue was fixed in 4% paraformaldehyde solution, embedded in paraffin, dehydrated, and sliced at 4 *μ*m. Some sections were stained with conventional HE, and the pathological changes of liver cells were observed under light microscope; some sections were subjected to immunohistochemistry.

### 3.5. RT-PCR

#### 3.5.1. Extraction of RNA from Liver Tissue

1. Take the liver tissue out of liquid nitrogen, place it in a mortar containing a small amount of liquid nitrogen, grind it, and replenish the liquid nitrogen in time, do not freeze the tissue, grind the tissue into a fine powder, add about 100 mg of tissue powder. Homogenize in a homogenizer containing Tripure for 2 minutes, and pipette repeatedly until the homogenization is complete, then transfer to a 1.5 mL EP tube, vortex at high speed for 2 minutes, and place at room temperature for 5 minutes.
2. Centrifuge at 12 000 g for 10 min at 4°C.
3. Aspirate the supernatant and place it in another centrifuge tube, and place it at room temperature for 10 minutes.
4. Add 0.2 mL of chloroform, mix vigorously for 20 seconds, and place at room temperature for 10 minutes.
5. Centrifuge at 12 000 g for 15 min at 4°C.
6. Centrifuge at 12 000 g for 10 min at 4°C.
7. Remove the supernatant, and wash the precipitate once with 75% ethanol.
8. 5% ethanol, wash again, 7500 g, 4°C centrifugation for 10 min. Remove the supernatant and place the centrifuge tube flat on a dust-free environment or on an ultraclean workbench. When there are no obvious droplets on the wall of the centrifuge tube, add 20uIDEPC-treated sterile double-distilled water to dissolve the RNA precipitate; the dissolved RNA is a colorless and cool liquid.

RETRACTED

#### 3.5.2. RT-PCR Reaction

The amplified product was analyzed by 2.0% agarose gel electrophoresis, and the size of the PCR amplified product was determined by DNA marker I. Chemi ImagerTMs 5500 gel imaging analyzer (Alpha Innotech) was used for grayscale analysis. The gray scale ratio is quantitative. Part of the reaction system in the PCR process is shown in Table 1.

### 3.6. Hepatocyte Detection

#### 3.6.1. Detection of Serum Alanine Aminotransferase (ALT) and Aspartate Aminotransferase (AST)

After intraperitoneal injection of D-GalN at 4, 8, 12, 16, 20, and 24 hours, 2 mice were taken from the control group, and 4 mice from the model group, and SIL Qianyu group were anesthetized with Sumianling. The eyeballs were removed and 2–3 mL of blood was taken. Centrifuge at 4°C (100 r/min) to collect serum, Hitachi-7110 automatic biochemical analyzer (provided by the laboratory of Provincial Hospital) to detect serum ALT and AST levels.

#### 3.6.2. MTT Method to Determine the Survival Rate of Liver Cells

1. Aspirate the culture solution and wash once with WME.
2. Add 0.1 mL of MTT-containing medium to each well, and incubate for 4 hours in a carbon dioxide incubator at 37°C and 5% carbon dioxide.
3. Add 0.15 mL DMSO to each well, shake and mix on a shaker to allow the reduction product to fully dissolve. After 10 minutes, the optical density (OD) value was measured on the enzyme-linked detector, and the detection wavelength was 492 nm.

RETRACTED

## 4. Results and Discussion

### 4.1. Serum ALT and AST Levels

After injection of CCI4, the serum ALT and AST of the model group increased gradually over time, reaching a peak at 20 hours (ALT 1544.5 ± 336.62; AST 2341.25 ± 433.01), which was significantly different from the normal control group (*p* < 0.05). Serum ALT and AST increased gradually after injury in the SIL Qianpu group, but they were significantly lower than the model group (*p* < 0.05). Serum ALT and AST levels in each group. All treatment groups had increased AST. After treatment for 4, 8, and 12 hours, there was no significant difference between each treatment group and the control group (*p* > 0.05). After 12 hours of treatment, the AST activity of the 4 mM, 10 mM, and 16 mM group was significantly different from the control group (*p* < 0.01); the difference between the 20 mM group and the control group was significant (*p* < 0.05); the difference between the 2 mM group and the control group was not significant (*p* > 0.05). After treatment for 24 hours, the AST content of 2 mM, 4 mM, 10 mM, and 20 mM group and the control group were not significantly different (*p* > 0.05); there was a significant difference between the 16 mM group and the control group (*p* < 0.05). Serum ALT and AST levels are shown in Table 2. The analysis of serum ALT levels is shown in Figure 2. The analysis of serum AST levels is shown in Figure 3.

After injection of CCl4, the mice in the model group lost their hair, were irritable, lacked appetite, and were lethargic, which were prolonged at any time, and the changes were gradually obvious. There was no obvious change in body weight. Two mice died at 22 hours of injury, and the fatality rate was 8.3%. The surface of liver cells in hepatitis mice is shown in Figure 4. The liver tissue sections of mice in the normal control group are shown in Figure 5.

### 4.2. Expression of NF-KB in Liver Tissue and Analysis of Promoting Liver Absorption

Normal liver cells do not express NF-KB, or only a small amount is expressed in the cytoplasm; NF-KB expression increases rapidly after injury, and reaches a peak (38.36 ± 4.75%) at 4 hours, and both cytoplasm and nucleus are expressed. As time passed by, the expression gradually decreased, and it was close to normal at 24 hours; the hepatocytes of the SIL Qianpre group also had different degrees of positive expression, but compared with the model group, they were all decreased in parallel comparison at each time (*p* < 0.05). The relative area percentage of NF-KB positive cells in the reference system in different phases of each group. The expression of NF-KB in each group is shown in Table 3. The expression analysis of NF-KB in each group is shown in Figure 6. The signal path of NF-KB is shown in Figure 7. The small intestinal food retention rate (%) of the model group was higher than that of the negative control group, which was statistically significant (*p*=0.024). The results show that silibinin relieves allergic symptoms by correcting the abnormal microecological environment of the intestinal tract of allergic children. Silybin can repair the intestinal barrier function by reducing the permeability of the small intestine, enhancing the specific mucosal immune response, and reducing the release of inflammatory mediators; silybin's lipopolysaccharide endotoxin, specific motif DNA, and other components can stimulate NF-KB, and other factors are released to induce Th0 cells to differentiate into Th1 cells, while inhibiting Th2 cell response to regulate Th1 and Th2, correcting Th1/Th2 imbalance, regulating the intestinal immune system, and reducing the incidence and severity of allergies.

RETRACTED

In addition, different concentrations of silybin were set to treat liver cells. At 3 hours, there was no significant difference between each treatment group and the control group (*p* > 0.05). After treatment for 6 hours, the NO content between the 4 mM, 10 mM, 16 mM group, and the control group was significantly different (<0.01), and the 2 mM, 20 mM group, and the control group were significantly different (*p* < 0.05). After 9 hours of treatment, the NO content in the 10 mM, 16 mM group, and the control group were significantly different (*p* < 0.05), and there was no statistical significance among the other groups. After 12 hours of treatment, there was a significant difference between the 20 mM group, the control group, and the 2 mM group (*p* < 0.05); there was no statistical significance among the other groups. After treatment for 24 hours, the NO content between the 4 mM, 10 mM, 16 mM group, and the control group was significantly different (*p* < 0.01); the 2 mM, 20 mM group, and the control group were significantly different (*p* < 0.05). The cell processing conditions of each group are shown in Table 4. The analysis of the cell processing results of each group is shown in Figure 8.

When silibinin was administered at 240 mg/kg at 10 minutes after modeling, only 1 mouse died. Silibinin has a good therapeutic effect, but when administered 20 minutes after modeling, the mortality rate of mice increased to 50%, and the therapeutic effect was significantly weakened. When administered at 40 min, silibinin basically has no therapeutic effect. This shows that after liver damage in mice, the earlier the administration of silibinin, the more effective it is. If the administration time is later, the therapeutic effect will be greatly reduced. This reminds us that, in the clinical treatment of patients with liver disease, medication should be given as soon as possible. If the best medication time is missed, other treatment options should be taken decisively.  Table 5 shows the death of mice administered at different times. The comparison between normal liver and pathological liver is shown in Figure 9.

RETRACTED

## 5. Conclusion

With the development of science and technology, the level of smart medical technology is getting higher and higher. Using modern smart medical methods, silybin is used for the treatment and protection of the liver. In this paper, mice are used as the experimental objects. After the animal model is established, the experiment is carried out in groups. Each group has 10 mice. The normal group and the model group are given 0.5% CMC-Na solution and the silibinin group is given SB/CMC-Na suspension, and the remaining groups of mice were given low, medium, and high doses of SB/CMC-Na suspension, respectively. After continuous infusion of the solution for 7 days, the mice were sacrificed and a serum sample was taken to observe the changes in their cell tissues. The experimental results show that silibinin has a significant effect on liver protection. This research is helpful to advance the research of silybin in liver protection.

## Figures and Tables

**Figure 1:** Molecular structure of silybin (http://alturl.com/nuy3b).

**Figure 2:** Analysis of serum ALT levels.

**Figure 3:** Analysis of serum AST levels.

**Figure 4:** Surface of liver cells in hepatitis mice (http://alturl.com/nt9n8).

**Figure 5:** Liver tissue sections of mice in the normal control group (http://alturl.com/9963e).

**Figure 6:** Expression analysis of NF-KB in each group.

**Figure 7:** Signal pathway of NF-KB (http://alturl.com/mgtxn).

**Figure 8:** Analysis of cell processing results in each group.

**Figure 9:** Comparison of normal liver and pathological liver (http://alturl.com/k9366).

**Table 1:** Part of the reaction system in the PCR process.

Reaction system	Dose (*μ*l)	Response parameters
AMV/Polymerase	10	45°C, 45 min
Buffer (5×)	1	95°C, 2 min
10 mM dNTP mixture	1	95°C, 30 min
AMV reverse transcriptase	1	52°C, 1 min
TNF-*α* sense primer	1	68°C, 2 min

**Table 2:** Serum ALT and AST levels.

Phase (h)	Control G		Model G		SIL peteated G	
	ALT	AST	ALT	AST	ALT	AST
4	32 ± 2.83	64 ± 1.41	127.3 ± 23.44	501.7 ± 8.02	55.67 ± 8.02	156.7 ± 9.07
8	34.5 ± 6.3	84 ± 11.31	136.3 ± 17.90	540 ± 46.36	69.3 ± 17.00	204.7 ± 23.25
12	28.5 ± 2.1	61.5 ± 9.19	358.75 ± 24.76	611.5 ± 57.32	104.75 ± 15.52	302.75 ± 14.01
16	31 ± 4.24	44.5 ± 3.54	1499.25 ± 378	1883.5 ± 336.58	392 ± 42.31	689 ± 81.67
20	32.5 ± 3.5	50.5 ± 19.0	1544.5 ± 336.6	2341.25 ± 433.0	450.75 ± 52.70	900.75 ± 118.0
24	30.5 ± 4.9	43.5 ± 6.36	11 82 ± 354.18	1421 ± 379.3	344 ± 53.01	660.25 ± 120.1

RETRACTED

**Table 3:** Expression of NF-KB in each group.

Group (h)	Control G	Model G	SIL G
4	2.27 ± 0.18	38.36 ± 4.75	21.44 ± 4.60
8	2.19 ± 0.40	21.13 ± 1.82	15.79 ± 1.83
12	2.10 ± 0.59	12.48 ± 0.81	9.51 ± 0.73
16	2.09 ± 0.31	8.62 ± 1.63	6.91 ± 1.09
20	1.96 ± 0.25	5.83 ± 0.67	4.53 ± 1.24
24	2.55 ± 1.24	4.10 ± 1.15	2.63 ± 0.61

**Table 4:** Cell processing in each group.

Group	3 hours	6 hours	9 hours	12 hours	24 hours
Control group	2.16 ± 0.98	2.95 ± 1.53	3.74 ± 0.75	4.95 ± 3.0	3.11 ± 1.22
2 mM group	2.87 ± 1.94	7.89 ± 2.25	8.77 ± 3.34	9.545 ± 4.67	9.51 ± 4.25
4 mM group	3.21 ± 1.21	9.01 ± 3.03	9.16 ± 3.93	13.43 ± 8.42	10.50 ± 2.47
10 mM group	4.313.37	9.12 ± 2.19	10.33 ± 0.85	15.90 ± 0.49	11.24 ± 0.54
16 mM group	4.33 ± 4.11	9.18 ± 1 .85	11.40 ± 0.23	16.96 ± 0.4.0	11.43 ± 0.81
20 mM group	3.94 ± 2.76	8.98 ± 3.01	9.17 ± 0.26	19.32 ± 4.08	9.92 ± 1.33

**Table 5:** Mortality of mice administered at different times.

Groups	Number of animals (*n*)	Number of dead animals (*n*)	Mortality rate (%)
Blank group	20	0	0
Model group	20	1	95
Silibinin low-dose administration group	20	0	0
Silibinin medium-dose administration group	20	0	0
Silibinin high-dose administration group	20	0	0

## Data Availability

Data sharing not applicable to this article as no datasets were generated or analyzed during the current study.
